The article "Imrecoxib Inhibits Paraquat-Induced Pulmonary Fibrosis through the NF-κB/Snail Signaling Pathway" was published in 2020. Journal: Comput Math Methods Med.

# Imrecoxib Inhibits Paraquat-Induced Pulmonary Fibrosis through the NF-*κ*B/Snail Signaling Pathway

**DOI:** 10.1155/2020/6374014

**Published:** 2020-10-13

**Authors:** Haihao Jin

**Affiliations:** Department of Traditional Chinese Medicine, Liuzhou People's Hospital, Liuzhou, 545000 Guangxi Zhuang Minority Autonomous Region, China

## Abstract

**Objective:**

In recent years, pulmonary fibrosis caused by paraquat poisoning is still concerned. However, no effective drugs have been developed yet to treat paraquat-induced pulmonary fibrosis. The aim of our research is to investigate whether imrecoxib can inhibit paraquat-induced pulmonary fibrosis and its possible mechanism.

**Methods:**

Extraction of primary pulmonary fibrosis cells (PPF cells) in vitro by the method of trypsin digestion. RT-qPCR and western blot were employed to measure the transcription level and protein expression of EMT related markers in paraquat-induced A549 cells. MTT, wound-healing, and Transwell experiments were used to verify the effect of imrecoxib on the proliferation, migration, and invasion of PPF and HFL1 cells.

**Results:**

Firstly, our results confirmed that paraquat can induce EMT and activate the NF-*κ*B/snail signal pathway in lung epithelial cell A549. Furthermore, experimental results showed that imrecoxib could repress the proliferation, migration, and invasion of PPF and HFL1 cells. Finally, our study found that imrecoxib can inhibit EMT of paraquat-induced A549 cells by the NF-*κ*B/snail signal pathway.

**Conclusion:**

Imrecoxib can inhibit EMT of paraquat-induced A549 cells and alleviate paraquat-caused pulmonary fibrosis through the NF-*κ*B/snail signal pathway. Therefore, imrecoxib is a drug worthy of study in the treatment of paraquat-induced pulmonary fibrosis.

## 1. Introduction

Human pulmonary fibrosis (PF), especially idiopathic pulmonary fibrosis (IPF), is a fatal and chronic disease that causes fibroblast proliferation and excessive deposition of relative protein, which in turn disrupts the lung structure and function and eventually leads to respiratory failure [1–3]. In recent years, the mortality of pulmonary fibrosis is increasing, but the current drugs have no obvious therapeutic effect [4, 5]. At present, the drugs used to treat pulmonary fibrosis are either ineffective or have too many side effects. For example, the drug nintedanib can be used to treat IPF, but it can cause great hepatotoxicity to patients. Clinically, pirfenidone can be used to treat mild or moderate idiopathic pulmonary fibrosis, but it has many side effects, such as skin photosensitivity, liver injury, vomiting, and gastrointestinal reaction. Using glucocorticoids, such as dexamethasone, to treat pulmonary fibrosis through anti-inflammation is a classic treatment, but it can cause serious side effects such as the liver and kidney dysfunction and osteoporosis [6–10]. Therefore, it is urgent to find a drug that can not only effectively treat pulmonary fibrosis but also produce fewer side effects on patients.

The article "Imrecoxib Inhibits Paraquat-Induced Pulmonary Fibrosis through the NF-κB/Snail Signaling Pathway" was published in 2020. Journal: Comput Math Methods Med.

Paraquat is a nonselective, contact, low pollution, low residue, broad-spectrum, and efficient herbicide, which is widely used in agricultural production. Pulmonary fibrosis is the main cause of death of paraquat poisoning. In recent years, pulmonary fibrosis caused by paraquat poisoning is still concerned. Many studies have proved that EMT is one of the main causes of paraquat induced pulmonary fibrosis and paraquat poisoning in humans and animals. Epithelial-mesenchymal transition (EMT) is a specific procedure, causing cells phenotypes transformed. It plays an indispensable function in embryonic, tissue reconstruction, cancer metastasis, inflammation, and many fibrotic diseases. Its obvious characteristics are the decrease of the expression of E-cadherin, the increase of vimentin, and the change of cells morphology. During fibrosis, an EMT-like process occurs [11, 12]. As a very important factor of EMT, NF-*κ*B can promote the release of a large number of inflammatory related factors, such as TNF-*α*, IL, and TGF-*β*. Many studies have shown that TGF-*β* is related to pulmonary fibrosis. For example, some studies have confirmed that doxycycline can regulate the balance between epithelial cells and mesenchymal cells and affect the TGF-*β* signal pathway to achieve the purpose of treating paraquat-induced pulmonary fibrosis [13]. The epithelial-to-mesenchymal transition of pulmonary fibrosis is induced through the TGF-*β*/smad signaling pathway [14]. Parthenolide is able to influence the level of EMT-related proteins and to treat pulmonary fibrosis by affecting the progression of pulmonary fibrosis through the NF-*κ*B/Snail signaling pathway [15]. Therefore, EMT, NF-*κ*B, and related inflammatory factors (TGF-*β*, TNF-*α*, and IL) are very important in the evaluation of pulmonary fibrosis.

Imrecoxib is a cyclooxygenase-2 (COX-2) inhibitor with anti-inflammatory effect, mainly used in the treatment of arthritis pain [16]. The drug was approved for marketing by the State Food and Drug Administration (SFDA) on May 20, 2011. Imrecoxib can not only inhibit inflammation and pain but also reduce the risk of gastrointestinal tract stimulation and cardiovascular injury [17]. The therapeutic effect of imrecoxib arthritis has been confirmed, but there are few studies on the effect of imrecoxib on pulmonary disease. There are research reports that cyclooxygenase-2 (COX-2) is associated with angiogenesis and lymphatic metastasis of NSCLC [18]. For example, celecoxib and nimesulide, as COX-2 inhibitors, can repress the progression of lung cancer [19, 20]. Only studies have shown that at the animal level, imrecoxib has a certain effect on lung adenocarcinoma cells by affecting the invasion and metastasis. However, there is no study on the effect of imrecoxib on pulmonary fibrosis. The purpose of this research is to study the effect of imrecoxib on pulmonary fibrosis and further study the mechanism.

The article "Imrecoxib Inhibits Paraquat-Induced Pulmonary Fibrosis through the NF-κB/Snail Signaling Pathway" was published in 2020. Journal: Comput Math Methods Med.

## 2. Materials and Methods

### 2.1. Reagents

Imrecoxib was acquired from Biofount Biotechnology Co., Ltd. (Beijing, China). The antibodies were all obtained from Abcam.

### 2.2. Isolation of Primary Pulmonary Fibrosis Cells

Mice treated with paraquat were killed, and their lungs were taken out and cut into small pieces. Then, we digested the lung samples with pancreatin and isolated the pulmonary fibrosis cells. Then, we cultured them and screened the primary pulmonary fibrosis (PPF) cells which can proliferate stably in vitro.

### 2.3. Cell Culture

HFL1 cells were originated from Shanghai Sixin Biotechnology Co., Ltd. HFL1 cells and isolated primary pulmonary fibrosis cells were cultured in DMEM medium containing 10% fetal bovine serum (FBS) in a sterile incubator at 37°C and in a 5% CO_2_ atmosphere. Human lung adenocarcinoma epithelial cell line A549 was cultured in RPMI-1640 medium.

### 2.4. Paraquat-Induced Lung Epithelial Cell A549 Assay

Lung adenocarcinoma epithelial cell A549 was inoculated in a 6-well plate and set to the control group and paraquat-induced group. The control group was cultured with normal RPMI-1640 medium, but the paraquat-induced group was cultured in RPMI-1640 medium with 20 *μ*mol/L paraquat. A549 cells were cultured for 5 days at 37°C and in a 5% CO_2_ condition. On the third day, the medium of the control group was substituted with fresh medium, and the medium of the paraquat-induced group was substituted with fresh culture medium with 20 *μ*mol/L paraquat. A549 cells were cultured until the 5th day.

### 2.5. MTT Assay

HFL1 cells and PPF cells with imrecoxib or without imrecoxib were inoculated in 96-well plates and cultured certain time at 37°C and in a 5% CO_2_ condition. After 24 or 48 hours, MTT reagent was put in, and then the cells were maintained for another 4-6 hours in dark. Thereafter, DMSO was added to react for 10 minutes, and the 96-well plates were shaken sufficiently to dissolve the crystal in the cells. Then, at the wavelength of 570 nm, the light absorption value of each well was measured by Microplate Reader. The cell viability of the control group and the imrecoxib-treated group was calculated by graphpad prism 5 software.

The article "Imrecoxib Inhibits Paraquat-Induced Pulmonary Fibrosis through the NF-κB/Snail Signaling Pathway" was published in 2020. Journal: Comput Math Methods Med.

### 2.6. Wound-Healing Assays

Mark with a marker pen at the bottom of sterile 6-well plate. Then, HFL1 or PPF cells were added in a sterile 6-well plate and cultured overnight in an incubator. When the cell confluency was close to 100%, a straight line was scraped on the cell surface with a sterile pipette tips. Then, the cells were cultured in serum-free medium with or without imrecoxib for 24 hours, and the 6-well plate were taken at 0, 6, 12, and 24 hours, respectively, and the migration distance of cells in different groups at different time points was recorded.

### 2.7. Transwell Assay

Prepare Matrigel diluted with serum-free medium in advance, put it into the upper chamber of Transwell, and then add the cell suspension with imrecoxib or without imrecoxib after the coagulation of Matrigel. Serum-free medium was put into the upper part, and medium containing serum was put into the lower chamber. Culture the cells in the condition of 37°C, 5% CO_2_ for 24 hours. Transwell chamber was removed and fixed with glutaraldehyde, and then the excess glutaraldehyde solution was washed by PBS. Thereafter, cells were stained by hexamethylpararosaniline and wiped off the upper cells with cotton swabs. Finally, the invading cells were photographed under a microscope, and the number of invading cells in different group was recorded.

### 2.8. Real-Time Quantitative PCR Assay

Prepare treated or untreated cell samples and extract RNA with Trizol reagent. After the RNA concentration was determined, the PCR reaction system was formulated based on the protocol of the fluorescent RT-qPCR kit, and the PCR cycle was carried out. The sequences of snail are F: 5′-TCGGAAGCCTAACTACAGCGA′, R: 5′-AGATAGCATTGGCAGCGAG-3′. The primer sequences of *β*-actin are F: 5′-CCTGTACGCCAACACAGTGC-3′, R: 5′-ATACTCCTGCTTGCTGATCC-3′; the primer sequences of E-cadherin are F: 5′-TGGACAGGGAGGATTTTGAG-3′, R: 5′-ACCTGAGGCTTTGGATTCCT-3′. The primer sequences of vimentin are F: 5′-GAGAACTTTGCCGTTGAAGC-3′, R: 5′-CTCAATGTCAAGGGCCATCT-3′. The reaction conditions were as follows: 95°C predenaturation for 10 min, 95°C for 10 s, 60°C for 60 s, and 40 cycles were performed. Three replicate wells were set for each gene, and the gene expression was calculated using the 2^–*ΔΔ*Ct^ method. The experiment was repeated three times.

### 2.9. Western Blot Assay

The treated or untreated cells were placed on ice and treated with RIPA lysate for 20 minutes. And the cells were collected in EP tubes and centrifuged to obtain protein samples. All protein samples were adjusted to the same concentration, and the polyacrylamide gel electrophoresis step was performed to separate the proteins with different molecular weights. Then, the protein on the gel was transferred to the nitrocellulose (NC) film. The hydrophobic binding sites on the nitrocellulose film were blocked with 5% BSA. After blocking, the membrane was added with primary antibody NF-*κ*B (Abcam, 1: 1000), snail (Abcam, 1: 500), and GAPDH (Abcam, 1: 2000) and incubate at 4°C overnight. Then, added the corresponding horseradish peroxidase labeled secondary antibody to react in the dark for 1 hour. Finally, the protein was detected and photographed according to the operation of the BeyoECL Plus chemiluminescence kit (Beyotime).

The article "Imrecoxib Inhibits Paraquat-Induced Pulmonary Fibrosis through the NF-κB/Snail Signaling Pathway" was published in 2020. Journal: Comput Math Methods Med.

### 2.10. Statistical Analysis

All the recorded data are analyzed by SPSS19.0 software, and all the data are recorded by means of mean ± SD. A *P* value less than 0.05 is considered statistically significant.

## 3. Results

### 3.1. Paraquat Can Induce EMT in A549 Cells

To investigate the effect of paraquat on epithelial-mesenchymal transitions of A549 cells, we divided the cells of A549 into the control group and paraquat-induced group. The RNA of two groups of A549 cells was extracted for the RT-qPCR assay, and the content of E-cadherin and vimentin in the two groups of A549 cells was determined by western blot. The data demonstrated that the expression of E-cadherin in the paraquat-induced group was much lower, but on the contrary, the expression of vimentin was significantly higher (Figures 1(a)–1(c)). These results indicated that paraquat can inhibit the expression of E-cadherin in A549 cells, while promote the vimentin expression, that is paraquat can induce the epithelial-mesenchymal transitions of A549 cells.

### 3.2. Paraquat Can Induced the NF-*κ*B/Snail Signaling Pathway in Lung Epithelial Cell A549

NF-*κ*B/snail is a very important signaling pathway in the EMT process. In order to study the efficacy of paraquat on the NF-*κ*B/snail signaling pathway in A549 cells, we extracted mRNA and protein from the control group and the paraquat-induced group of A549 cells, respectively, and performed RT-qPCR and western blot assay to study the effects of paraquat on mRNA and protein of NF-*κ*B and snail in A549 cells. Our data showed that the level of mRNA of NF-*κ*B and snail in A549 cells of the paraquat-treated group was significantly higher than that of the control group (Figures 2(a) and 2(b)). Furthermore, the results of western blot also demonstrated that the protein expression is a consistent trend with mRNA (Figure 2(c)). The above results all confirmed that paraquat could induce the NF-*κ*B/snail signaling pathway in A549 cells.

### 3.3. Imrecoxib Can Inhibit the Proliferation and Migration of PPF Cells

Primary pulmonary fibrosis cells (PPF cells) are a kind of cells with mesenchymal phenotype, which are extracted from the lungs of paraquat-treated mice. PPF cells were set into two groups: control group and imrecoxib-treated group. According to the results of MTT, the cell viability of PPF cells treated with imrecoxib was lower than that without imrecoxib (Figure 3(a)). The results showed that imrecoxib could inhibit the proliferation of PPF cells. Besides, the findings of cell wound-healing assays and transwell revealed that the invasion and migration ability of PPF cells in the imrecoxib-treated group was much weaker when compared with THE control group. In other words, imrecoxib can significantly inhibit the invasion and migration ability of PPF cells (Figure 3(b)). The above experiments showed that imrecoxib can suppressed the proliferation, migration, and invasion functions of PPF cells.

The article "Imrecoxib Inhibits Paraquat-Induced Pulmonary Fibrosis through the NF-κB/Snail Signaling Pathway" was published in 2020. Journal: Comput Math Methods Med.

### 3.4. Imrecoxib Can Inhibit the Proliferation and Migration of HFL1 Cells

HFL1 cell is a human fetal pulmonary fibrosis cell with mesenchymal phenotype. Similar to the result of imrecoxib on PPF cells, MTT test showed that imrecoxib could inhibit the proliferation of HFL1 cells (Figure 4(a)), and the wound-healing test showed that imrecoxib could inhibit the migration of HFL1 cells (Figure 4(b)). These results indicated that the drug imrecoxib can also inhibit the proliferation and migration HFL1 cells.

### 3.5. Imrecoxib Can Inhibit Paraquat-Induced EMT in Lung Epithelial Cell A549

We further studied the effect of imrecoxib on EMT of A549 cells induced by paraquat. We set three groups: control group (untreated A549 cells), imrecoxib-treated group (paraquat-induced A549 cells were treated with imrecoxib), paraquat-induced group (paraquat-induced A549 cells).We measured the content of E-cadherin and vimentin by western blot in three groups, respectively. The results displayed that the E-cadherin level of A549 cells in the control group was the highest, followed by that in the imrecoxib-treated group and the lowest in the paraquat-induced group. In contrast to the E-cadherin expression, the vimentin expression of A549 cells in the control group was the lowest, the imrecoxib-treated group was the second highest, and the vimentin expression of A549 cells in the paraquat-induced group was the highest (Figure 5(a)). The above experimental results show that imrecoxib can affect the expression of EMT-related proteins; specifically, imrecoxib can inhibit paraquat-induced EMT in lung epithelial cell A549.

### 3.6. Imrecoxib Can Inhibit Paraquat-Induced the NF-*κ*B/Snail Signaling Pathway in Lung Epithelial Cell A549

Our experiments have confirmed that paraquat can induce the NF-*κ*B/snail signal pathway of A549 cells. What we need to study next is the relationship between imrecoxib and the signal pathway. We divided A549 cells into three groups: control group (untreated A549 cells), imrecoxib-treated group (paraquat-induced A549 cells were treated with imrecoxib), paraquat-induced group (paraquat-induced A549 cells). First, we measured the miRNA transcription level of NF-*κ*B and snail of A549 cells in three groups by RT-qPCR. The results displayed the mRNA level of NF-*κ*B and snail in paraquat-induced group was the highest, that of the mRNA level of the control group was the lowest, and that of the mRNA level in the imrecoxib-treated group was between that of the control group and paraquat-induced group. The above results confirmed that imrecoxib could suppress the mRNA level of NF-*κ*B and snail in paraquat-induced A549 cells (Figure 6(a)). We further studied the effect of imrecoxib on NF-*κ*B and snail protein in paraquat-induced A549 cells by western blot, which showed that the two protein content was the highest in the paraquat-induced A549 cell group and the lowest in A549 cells of the control group. The two protein levels in the imrecoxib-treated group were between the control group and paraquat-induced group. Our data showed that imrecoxib could affect the expression of NF-*κ*B and snail protein in paraquat-induced A549 cells; specifically, imrecoxib could inhibit the expression of NF-*κ*B and snail protein in paraquat-induced A549 cells (Figure 6(b)). The above experimental results confirmed that imrecoxib can not only inhibit the transcription levels of NF-*κ*B and snail in paraquat-induced A549 cells but also can inhibit the protein expression levels.

The article "Imrecoxib Inhibits Paraquat-Induced Pulmonary Fibrosis through the NF-κB/Snail Signaling Pathway" was published in 2020. Journal: Comput Math Methods Med.

## 4. Discussion

Imrecoxib is a kind of drug that can moderately inhibit COX-2 to play an anti-inflammatory role. It has a good inhibition of inflammation and pain, but also reduces the chance of gastrointestinal tract stimulation and cardiovascular damage [16]. At present, only a few studies have confirmed that imrecoxib can repress the invasion and metastasis of NSCLC, but the mechanism is not clear. It is only speculated that the possible mechanism is to inhibit the inactivation of PTEN protein, interfere with PI3K/Akt signal transduction, block cell cycle in the G1 phase, or promote apoptosis [21]. But at present, there is almost no research on imrecoxib in the pulmonary fibrosis field. For the sake of research on the effect of imrecoxib on pulmonary fibrosis cells, we carried out MTT and wound-healing assays. The current experimental results demonstrated that imrecoxib can inhibit the proliferation, migration, and invasion of PPF and HFL1 cells.

The article "Imrecoxib Inhibits Paraquat-Induced Pulmonary Fibrosis through the NF-κB/Snail Signaling Pathway" was published in 2020. Journal: Comput Math Methods Med.

The main cause of paraquat poisoning is that it can cause pulmonary fibrosis. There are many studies on the mechanism of paraquat inducing pulmonary fibrosis. EMT plays an important role in paraquat-induced pulmonary fibrosis [22]. It has been confirmed that paraquat can activate the Wnt/*β*-Catenin signal pathway and then induce EMT of type II alveolar epithelial cells, which is mainly manifested as the decrease of the E-cadherin expression and the increase of the vimentin expression [23]. More and more evidence showed that cytokines play an essential role in EMT. For example, transforming growth factor *β* (TGF-*β*) is considered to be one of the main cytokines in paraquat-induced pulmonary fibrosis, and it is also a research hotspot of scholars at home and abroad. Paraquat can induce EMT and active TGF-*β*/Smad signal pathway [24, 25]. Our results showed that paraquat can activate EMT by inhibiting E-cadherin mRNA and protein expression of A549 cells and promoting vimentin mRNA and protein expression. And our experimental results indicated that imrecoxib can reduce the inhibition on E-cadherin and promotion on vimentin in paraquat-induced A549 cells and then inhibit the EMT activated by paraquat, so as to treat paraquat-induced pulmonary fibrosis.

Moreover, studies have shown that paraquat can activate inflammatory related factors including TNF*α*, NF-*κ*B, interleukin 1*β*, and IL-6, which in turn contribute to the development of pulmonary fibrosis [26]. NF-*κ*B is a crucial transcription regulator, which plays an extremely important function in the process of inflammation, immunity, and apoptosis. In addition, NF-*κ*B is also involved in the occurrence and development of fibrosis by regulating transcription factors related to fiber growth, such as PDGF and TGF-*β*1. The expression product of the snail gene is a transcription factor that plays an important effect in the process of EMT. We evaluated the expression of NF-*κ*B and snail mRNA and protein in paraquat-induced A549 cells. The results showed that paraquat could activate the transcription of NF-*κ*B and snail mRNA and protein in A549 cells. Moreover, we further evaluated the effect of imrecoxib on NF-*κ*B and snail in paraquat-induced A549 cells. The results proved that the level of miRNA transcription and protein expression of NF-*κ*B and snail in A549 cells activated by paraquat was alleviated after treatment with imrecoxib. These results suggest that imrecoxib can attenuate the activation of NF-*κ*B and snail induced by paraquat and thus play a role in the treatment of pulmonary fibrosis. The NF-*κ*B pathway activates the snail expression through transcriptional and posttranslational mechanisms. Moreover, NF-*κ*B can be bind to the promoter of snail, further to increase the transcription of the snail. Therefore, imrecoxib can inhibit paraquat-induced pulmonary fibrosis by inhibiting the NF-*κ*B/snail signal pathway.

The article "Imrecoxib Inhibits Paraquat-Induced Pulmonary Fibrosis through the NF-κB/Snail Signaling Pathway" was published in 2020. Journal: Comput Math Methods Med.

To sum up, we first established the A549 cell model induced by paraquat and confirmed that paraquat can change the transcription and protein expression ability of E-cadherin and vimentin in A549 cells at the level of gene transcription and protein expression, indicating that paraquat can activate the EMT of A549 cells. Then, by measuring the mRNA and protein expression of NF-*κ*B and snail in A549 cells induced by paraquat, we proved that paraquat activated the NF-*κ*B/snail signal pathway in A549 cells. Next, we assessed the influence of imrecoxib on PPF and HFL1 cells. The results showed that imrecoxib could suppress the proliferation and migration of PPF and HFL1 cells. Finally, we found that imrecoxib can activate the EMT in A549 cells induced by paraquat, accompanied by the activation of the NF-*κ*B/snail signal pathway. Our study shows that imrecoxib are expected to be an effective drug for paraquat-induced pulmonary fibrosis. Therefore, our research not only provides a new idea to treat paraquat-induced pulmonary fibrosis but also intends the treatment methods of imrecoxib. However, the effect or mechanism of imrecoxib in treating pulmonary fibrosis needs further study.

## 5. Conclusion

Our results confirm that imrecoxib can inhibit EMT of paraquat-induced A549 cells and alleviate paraquat-induced pulmonary fibrosis through the NF-*κ*B/snail signal pathway.

## Figures and Tables

**Figure 1:** mRNA and protein expression of EMT markers in paraquat-induced lung epithelial cell A549. (a). The mRNA level of E-cadherin in A549 cells of the control group and paraquat-induced group was measured by the RT-qPCR method. (b). The mRNA level of vimentin in A549 cells of the control group and paraquat-induced group was measured by the RT-qPCR method.(c). The protein expression of E-cadherin and vimentin in A549 cells of the control group and paraquat-induced group was measured by western blot. ^∗∗∗^*P* < 0.001.

**Figure 2:** mRNA and protein expression of NF-*κ*B and snail in paraquat-induced lung epithelial cell A549. (a). The mRNA level of NF-*κ*B in A549 cells of the control group and paraquat-induced group was measured by the RT-qPCR method. (b). The mRNA level of snail in A549 cells of the control group and paraquat induced group was measured by the RT-qPCR method. (c). The protein expression of NF-*κ*B and snail in A549 cells of the control group and paraquat-induced group was measured by the western blot method. ^∗∗^*P* < 0.01.

The article "Imrecoxib Inhibits Paraquat-Induced Pulmonary Fibrosis through the NF-κB/Snail Signaling Pathway" was published in 2020. Journal: Comput Math Methods Med.

**Figure 3:** Effects of imrecoxib on the proliferation and migration and of PPF cells in vitro. (a) The effect of imrecoxib on the proliferation ability of PPF cells was measured by the MTT assay. (b). The effect of imrecoxib on the migration ability of PPF cells was measured by the scratch test. (c) The effect of imrecoxib on the invasion ability of PPF cells was measured by transwell. ^∗∗^*P* < 0.01; ^∗∗∗^*P* < 0.001.

**Figure 4:** Effects of imrecoxib on the proliferation and migration of HFL1 cells in vitro.(a) The effect of imrecoxib on the proliferation ability of HFL1 cells was measured by the MTT assay. (b) The effect of imrecoxib on the migration ability of HFL1 cells was measured by the scratch test.^∗∗∗^*P* < 0.001.

**Figure 5:** The effect of imrecoxib on the mRNA expression of E-cadherin and vimentin in paraquat-induced A549 cells was assessed by RT-qPCR. #*P* < 0.05; ^∗∗^*P* < 0.01; ^∗∗∗^*P* < 0.001.

**Figure 6:** The effect of imrecoxib on NF-*κ*B and snail mRNA transcription and protein expression in paraquat-induced A549 cells. (a, b) The effect of imrecoxib on the mRNA level of NF-*κ*B and snail in paraquat-induced A549 cells was determined by the RT-qPCR method. (c) The effect of imrecoxib on the protein expression of NF-*κ*B and snail in paraquat-induced A549 cells was measured by the western blot method. **#***P* < 0.05; ^∗∗^*P* < 0.01.

## Data Availability

All the data could be provided if qualified authors required it.
